The article "Cost Control of Mining Personnel Based on Wireless Communication Network from the Perspective of Operations Research" was published in 2022. Journal: Comput Intell Neurosci.

# Cost Control of Mining Personnel Based on Wireless Communication Network from the Perspective of Operations Research

**DOI:** 10.1155/2022/9932603

**Published:** 2022-01-10

**Authors:** Hongyi Wang, Meichang Zhang

**Affiliations:** ^1^Management Science and Engineering, Liaoning Technical University, Fuxin 123000, China; ^2^Mining Engineering, Liaoning Technical University, Fuxin 123000, China

## Abstract

The sublevel caving method without sill pillar is used to improve the cost of mining. The analysis is performed according to unique geographical environment and the current mining technology of the mine. The wireless communication network is used to budget and control the work cost of mining. Simulation operation about unit explosive dosage, fan-shaped deep hole interval, hole bottom distance, and collapse step distance is performed. Experiments have shown that budget and control of the cost of mining workers with wireless communication technology can manage mining data and guide the design of mining data.

## 1. Introduction

The cost control by mining personnel is a relatively complex system. Due to the continuous changes in the production of mining factories, the cost control of mining personnel needs to consider the overall balance of different links, continuity, and uncertainty, in order to carry out effective identification and optimization, and control the cost of mining personnel of mine engineering. With the rapid development of science and technology, digitization and visualization technology have been widely used in various fields. As the main component of the mine, development plan for cost control of mining personnel is needed, digitizing and visualizing the mining activities, timely and accurately recording and expressing the engineering changes in the mine pit, and improving the mining level and work efficiency [1–3].

The construction of an integer model is used to optimize the location of fans in the network and the selection of structures in this paper. The cost of ventilation is normalized to minimize it. For the same problem, the nonlinear unmixed model covers special constraints and branch constraints, which are the basis for semiconstrained design, and optimizes the answer.

## 2. Establishment of Operational Research Model

The constrained flow network problem only includes the best deployment location of personnel and building selection to allocate personnel to all predetermined network branches [4–6]. The problem of nonholonomic constraints of the network will face a dual task. In addition to determining the best placement of personnel and the choice of structures, it is also necessary to control the people flowing into unclear branches.

### 2.1. Constrained Flow Network Problem

Because the distribution of personnel in the network is known, the constrained condition conditions do not need to be discussed, and then the objective function of this problem can be expressed by formula (3), and its constrained conditions are

(1) $$\begin{array}{c} \left\{\begin{array}{c} \sum_{j=1}^{b}\left(R_{j}\left|Q_{j}\right|Q_{j}+HR_{j}-HN_{j}-HF_{j}\right)=0,\\ HR_{j},HN_{j}\geq 0,j=1,\ldots ,b. \end{array}\right. \end{array}$$

Obviously, this is a nonlinear programming model, which is transformed into a linear programming model by introducing bivariate *Y*_*j*_ and the objective function is transformed by obtaining this value *Y*_*j*_.

(2) $$\begin{array}{c} Y_{j}=\left\{\begin{array}{cc} 1, & HF_{j}>0,\\ 0, & \text{other,} \end{array}\right.\;,C_{p}Q_{j}=a_{j},\\ \text{minimize Z}=\sum_{j\in L}a_{j}HF_{j}+\sum_{j\in L}C_{j}Y_{j}. \end{array}$$

The constrained conditions are

(3) $$\begin{array}{c} \left\{\begin{array}{c} \sum_{j=1}^{b}b_{ij}\left(R_{j}\left|Q_{j}\right|Q_{j}+HR_{j}-HN_{j}-HF_{j}\right)=0,\\ HR_{j},HF_{j}\leq 0,j=1,\ldots ,b,\\ HF_{j}\leq d_{j}Y_{j},j\in L,\\ Y_{j}=\left(0,1\right). \end{array}\right. \end{array}$$

In the formula, *d*_*j*_=max*HF*_*j*_. When *HF*_*j*_ ≠ 0, *Y*_*j*_=1; when *HF*_*j*_=0, *Y*_*j*_=0 时. So when *Y*_*j*_=1, *Y*_*j*_=0, and a larger value may appear in *Z*.

### 2.2. Half Constrained Flow Network Problem

Assume that the minimum value *L*_*j*_ and maximum values *U*_*j*_ of branchers, respectively, flow to ambiguous branchers and are represented by the objective function [7].

(4) $$\begin{array}{c} \text{MinZ}=\sum_{j=1}^{L}C_{j}Q_{j}HF_{j}+\sum_{j=1}^{L}C_{j}. \end{array}$$

The constrained conditions are

(5) $$\begin{array}{c} \left\{\begin{array}{c} \sum_{j=1}^{b}a_{ij}Q_{j}=0,\\ \sum_{j=1}^{b}b_{ij}\left(R_{j}\left|Q_{j}\right|Q_{j}+HR_{j}-HN_{j}-HF_{j}\right)=0,\\ L_{j}\leq Q_{j}\leq U_{j},\\ HR_{j}\geq 0,\\ X_{j}=\left(0,1\right),\\ Q_{j}HF_{j}\geq P_{j},X_{j}=1,\\ Q_{j}HF_{j}=P_{j},X_{j}=0,\\ j=1,\ldots ,b, \end{array}\right. \end{array}$$

where *P*_*j*_ is the minimum power allowed on branch *j*.

It can be seen from the previously mentioned objective function and constrained conditions that they are all nonlinear. So we need to transform it into a linear programming. During the transformation, the decompression is first determined, and then, the solutions for each subset are established. All solutions need to form the elements that make up the aggregation *L* for *X*_*j*_. Finally, this nonlinear programming is a linear programming, and then, the best solution is selected. The specific method is verified in the following example.

## 3. Specific Application of Operations Research

Figure 1 is a cost network diagram of a miner. It is composed of nine branches and six nodes, and each wind resistance is constant. According to the specific situation, the personnel can be configured for seven minutes when branching. On 8, the structures are at branches 3, 5, and 8.

The distribution of personnel on each branch is shown in Table 1.

### 3.1. Problem Solving for Constrained Flow Network

We select the spanning tree {1, 2, 5, 6, 9}, and the matrix can be obtained *b*_*ij*_

(6) $$\begin{array}{c} b_{ij}=\left[\begin{array}{ccccccccc} 1 & 2 & 3 & 4 & 5 & 6 & 7 & 8 & 9\\ -1 & 1 & 0 & 1 & 0 & -1 & 0 & 0 & 0\\ 0 & 1 & 0 & 0 & 1 & 0 & 1 & 0 & 0\\ 1 & 0 & 0 & 0 & 0 & 1 & 0 & 1 & 1 \end{array}\right]. \end{array}$$

Then, the objective function can be expressed as

(7) $$\begin{array}{c} \min Z=C_{p}Q_{5}HF_{5}+C_{p}Q_{7}HF_{7}+C_{p}Q_{8}HF_{8}+C_{5}Y_{5}+C_{7}Y_{7}+C_{8}Y_{8}. \end{array}$$

The constrained conditions are

(8) $$\begin{array}{c} \left\{\begin{array}{c} -R_{1}Q_{1}^{2}+R_{2}Q_{2}^{2}+R_{4}Q_{4}^{2}-R_{6}Q_{6}^{2}=0,\\ R_{1}Q_{1}^{2}-R_{2}Q_{2}^{2}+R_{3}Q_{3}^{2}+HR_{3}-R_{5}Q_{5}^{2}-HR_{5}+HF_{5}=0,\\ R_{2}Q_{2}^{2}+R_{5}Q_{5}^{2}+HR_{5}-HF_{5}+R_{7}Q_{7}^{2}-HF_{7}=0,\\ R_{1}Q_{2}^{2}+R_{6}Q_{6}^{2}+R_{8}Q_{8}^{2}-HF_{8}=0,\\ HF_{5}\leq d_{5}F_{5},\\ HF_{7}\leq d_{5}F_{7},\\ HF_{8}\leq d_{5}F_{8},\\ Y_{j}=\left(1,0\right),\;j=5,7,8,\\ HR_{j}\geq 0,\;j=3,5,8,\\ HR_{j}\geq 0,\;j=5,7,8. \end{array}\right. \end{array}$$

After calculation, the best solution is to set up two personnel on branches 7 and 8, respectively, where the wind pressure on branch 7 is 11330.6 Pa, 840.8 Pa of which is shared by branch 8. The main auxiliary equipment is set on branch 3.

The best solutions are usually difficult to be found for the multifunctional optimization problems. Most of them adjust each target in a balanced manner and meet the requirements based on the problem to obtain the best balanced solution with certain accuracy and practical significance. Here, the decisive objective function and constraint conditions in the problem are shown. Fuzzy theory is combined with intelligent algorithms to solve chaotic optimization problems. The dark color of more than one thousand targets is most suitable for the best dextrin of the basic thousand single targets. In the fuzzy set of the optimal solution of each target, the solution of each target is satisfied as much as possible.

(1) The objective function of the formula MOP problem is complex and only provides a very large membership function. On the premise of satisfying the constraints as much as possible, the larger the objectives, the better, and there is an upper limit but no lower limit. The upper limit is the best value for each single goal optimization [8–10]. Therefore, the ray shape is selected as the correlation function for each target.

(9) $$\begin{array}{c} \mu \left(f_{k}\left(X\right)\right)=\left\{\begin{array}{c} 1,f_{k}\left(X\right)>c_{01},\\ \frac{f_{k}\left(X\right)-c_{0k}+\delta_{0k}}{\delta_{0k}},c_{0k}-\delta_{0k}<f_{k}\left(X\right)\leq x_{0k},\\ 0,f_{k}\left(X\right)\leq c_{0k}-\delta_{0k}. \end{array}\right. \end{array}$$

In the formula, *μ*(*f*_*k*_(*X*)) specifies the membership function *f*_*k*_(*X*) of the target. The target value *f*_*k*_(*X*) for the target optimization of the target monomer *c*_0*k*_. This is the added value of target *δ*_0*k*_ accepted by policy makers, and it is determined by scaling to a certain extent on the basis of optimizing the target value into a single target (Figure 2).

The specific solution steps of the wireless communication network method are as follows:

*Step 1.* Use the following wireless communication network algorithm to find the optimal solution to the constraints of each single-objective function:
  (10) $$\begin{array}{c} \left\{\begin{array}{c} \max f_{i}\left(X\right),i=1,2,\ldots ,p,\\ g_{i}\left(X\right)\leq 0,i=1,2,\ldots ,m,\\ h_{j}\left(X\right)=0,j=1,2,\ldots ,l. \end{array}\right. \end{array}$$
Find the optimal solution of the constraint of the previously mentioned objective function.
*Step 2.* Stretch each single target value to a certain extent; that is, determine the added value
*Step 3.* The fuzzy of each objective function, that is, the function that determines the degree of membership of each objective function, is as follows:
  (11) $$\begin{array}{c} \mu \left(f_{k}\left(X\right)\right),k=1,2,\ldots ,p. \end{array}$$
Define the satisfaction degree of all membership functions as
  (12) $$\begin{array}{c} \lambda =\min\left\{\mu \left(f_{i}\left(X\right)\right),\mu \left(f_{2}\left(X\right)\right),\ldots ,\mu \left(f_{p}\left(X\right)\right)\right\}. \end{array}$$
*Step 4.* Substitute *c*_0*k*_*δ*_0*k*_ into (3) to obtain expression of *p* membership function.
*Step 5.* Based on the max-min law of the fuzzy set theory, the maximum satisfaction degree method is used to convert the multiobjective problem into a single-objective nonlinear problem. The mathematical model is as follows:
  (13) $$\begin{array}{c} \left\{\begin{array}{c} \max\lambda ,\\ f_{1}\left(X\right)-\delta_{01}\lambda \geq c_{01}-\delta_{01},\\ \cdots \\ f_{k}\left(X\right)-\delta_{0k}\lambda \geq c_{0k}-\delta_{0k},\\ \cdots \\ f_{p}\left(X\right)-\delta_{0p}\lambda \geq c_{0p}-\delta_{0p},\\ 0\leq \lambda \leq 1,\\ g_{i}\left(X\right)\leq 0,i=1,2,\ldots ,m,\\ h_{j}\left(X\right)=0,j=1,2,\ldots ,l. \end{array}\right. \end{array}$$
*Step 6.* The wireless communication network algorithm is applied to solve the previously mentioned single-objective fuzzy optimization model and find the optimal value of each objective function under a given satisfaction degree (90%).

### 3.2. Problem Solving for Half Constrained Flow Network

The personnel on branches 3, 4, and 7 are known to be 18.00 m^3^/s, 20.00 m^3^/s, and 35.00 m^3^/s, and a new matrix *a*_*ij*_ can be obtained.

(14) $$\begin{array}{c} a_{ij}=\left[\begin{array}{ccccccccc} 1 & 2 & 3 & 4 & 5 & 6 & 6 & 8 & 9\\ -1 & 1 & 0 & 1 & 0 & 1 & 0 & 0 & 0\\ 1 & -1 & 1 & 0 & -1 & 0 & 0 & 0 & 0\\ 0 & 1 & 0 & 0 & 0 & 0 & 1 & 0 & 0\\ 1 & 0 & 0 & 0 & 0 & 1 & 0 & 1 & 0 \end{array}\right]. \end{array}$$

We define the personnel of branches 7 and 8 as surface personnel and branch 5 as a candidate for underground personnel. The objective function is

(15) $$\begin{array}{c} \min Z=Q_{5}HF_{5}+aHF_{7}+Q_{8}HF_{8}. \end{array}$$

Suppose *Z*_1_=(*Q*_*i*_+*HF*_8_)/2, *Z*_2_=(*Q*_8_ − *HF*_8_)/2 and then introduce nonnegative special variables *λ*_*k*_, *u*_*k*_, and *v*_*k*_, so that ∑_*k*_*λ*_*k*_=0,  ∑_*k*_*u*_*k*_=0,  ∑_*k*_*v*_*k*_=0. Then, *Z*_1_, *Z*_2_, and *Q*_8_ can be expressed as *Q*_8_=∑_*K*_*λ*_*k*_*Q*_8*k*_,  *Z*_1_=∑_*k*_*u*_*k*_*Z*_1*k*_,  *Z*_2_=∑_*k*_*v*_*k*_*Z*_2*k*_. Then, the previously mentioned problem can be transformed into linear programming, and its objective function is

(16) $$\begin{array}{c} \min Z=Q_{5}HF_{5}+Q_{7}HF_{7}+\sum_{k}u_{k}Z_{1k}^{2}-\sum_{k}v_{k}Z_{2k}^{2}. \end{array}$$

After calculation, the wind pressure on branch 7 is 840.88 Pa, the wind pressure shared by branch 8 is 113.6 Pa, and the wind pressure on branch 5 is 374.35 Pa.

## 4. The Basic Function and Innovation of the Cost Control System for Mining Personnel

A simulation model of the mine's in-pit visual production system is built according to the actual situation of the specific mine at first, and simulation operation is performed after the model is verified and confirmed. The in-pit production process is observed dynamically in the mine. In addition, the operating status of each stage of the biological flow system of mine can be analyzed in real time. The development logic program of the dynamic optimization policy decision system for the three-dimensional dynamic visualization of underground mine engineering is as follows [11, 12].

1. Information about mine production systems is collected for specific mines. It contains the parameters related to the tunnel formation system: the logistics process, production capacity, and technical parameters and capabilities of related equipment in the production system of coal mining, ventilation, transportation, drainage, and so on.
2. Statistical analysis and integration is performed for the previously mentioned collected data related to the cost control system for underground mining personnel.
3. Analyze the various influencing factors of mine production, define the boundaries of the mine logistics system, and divide the subsystems according to the functions of the logistics process of mine.
4. On the basis of a large number of field investigations and statistical analysis, the statistical rules and parameters of each part of the mining system are determined.
5. Through the mine layout system and production system of the built mine, the connection and conversion relationship between the various subsystems of the mine production is found out, the integration capability of the various equipment of the mine production system and the logistics system is established, and a fully visualized underground mine model of mining personnel cost control system is built.
6. According to the simulation software of WITNESS, the cost control system model of the underground mining personnel of the mine is reasonably converted into a computer simulation model.
7. The reliability simulation of the simulation model was verified, the interference of random factors was eliminated, the simulation results were statistically analyzed, and unreasonable factors in the system were found.
8. The model is improved to make it more in line with the actual mine production system.
9. According to the actual production of mine, the simulation operation of the mine logistics system is carried out. According to the simulation results, the mine logistics system is rationally optimized and integrated, to apply the improvement plan to the mine production practice and compare the improved demonstration operation result with the actual mine production practice effect for evaluation.

Among them, the key issues in the development of the mining personnel cost control system are as follows.

1. Collect true information about mine production systems for specific mines: the parameters of the tunnel configuration system, coal mining, excavation, ventilation, transportation, drainage, and other logistics process, production capacity, and technical parameters and capabilities of related equipment
2. Import mine development engineering drawings (Figure 3) into the WITNESS system. The imported engineering drawings will be imported to the prebuilt system modules based on the actual underground mining personnel cost control system process (Figure 4: the mine underground mining personnel cost control system process) to build a simulation model of the mine's in-pit visual production system.
3. Perform the validity check of the simulation model of the in-pit visual production system in the mine. Transform the parameters of field survey and statistical analysis (including technical indicators such as underground logistics equipment capability, failure rate, repair rate, and other reliability indicators) into computer simulation models. Carry out simulation operation, analyze it combined with the actual logistics system operation, carry out validity check, and ensure the validity of the simulation system.

## 5. Realization of Cost Control of Mining Personnel

### 5.1. Projective Transformation

The functions of the wireless communication network-like calculation procedure library cannot directly generate arc surfaces. If the NURBS surface adopted cannot be correctly controlled, it cannot meet the need of explaining the lane. In addition, the complicated program leads to the low operation efficiency. In this study, an arched lane is made by adding a tangent plane. The arched lane is composed of two concentric cylinders with different radii and two concentric circular plates. Projective transformation is an important graphics conversion technique whose purpose is to define the view. The extra part outside the field of view is intercepted, and the final image is only the relevant part of the visual field.

In perspective projection, the projection close to the point is very large, the projection from the viewpoint is very small, and the projection that reaches the extreme point disappears and becomes the vanishing point. The projection is mainly used for meeting animation requests, visualization and other image display areas. In the mine mining intelligent analysis system, the proportional relationship between the alleys remains unchanged after the projection transformation for a more reasonable use of the relative spatial positions of different projects for the mining project layout of the mine.

### 5.2. Illumination Treatment

The illumination model of the algorithm is, for example, wireless communication network, radiation, ambient light, diffused light, specular light, and so on. The radiation is emitted directly from the object and is not affected by the light source. Ambient light is scattered multiple times from the light source through the environment, and light that cannot determine its direction is considered to come from all directions. The diffused light comes from a certain direction. It is brighter when it is perpendicular to the object than when it is tilted. After irradiating the object, it will be distributed evenly in all directions. Specular light comes from a specific direction and reflects in other directions.

The purpose of the illumination model is to make the generated graphic image be truly felt by performing complex calculations on normal, light sources, materials, and so on. The command to start the illumination model is glEnbale. LIGHTING), gDiscable (GL_LIGHTING) turn off the current light.

### 5.3. Plane Normal Vector

The calculation vector strictly represents the direction between multiple countries. Open GL needs to use the normal vector to calculate the angle of light irradiating the object. In order to generate a three-dimensional image, the normal vector of the object must be defined. The wireless communication network algorithm uses two functions to define the normal vector. The first function means the three component values of the normal vector, respectively, given by the function. Second, define a pointer with three elements. The wireless communication network does not provide a function of the corona calculation method. Therefore, it is necessary to create a corresponding program for the developer. The normal vector algorithm designed in this research is verified by actual data and is accurate and effective.

### 5.4. Integrated Implementation

The characteristics of the following aspects are mainly reflected in the research and development process.

1. In order to facilitate the development and use, this system adopts a modular design concept to construct a three-dimensional dynamic visualization system and related equipment modules for the engineering in the pit. Using this modular structure, different mines can be constructed: underground laborers and three-dimensional dynamic visualization simulation to determine the needs of the system.
2. Regarding the logistics process and flow of the simulation system model, in the CAD engineering drawing of the actual mine production system, such as the introduction of mine development and mining plan, the structure configuration and construction of the simulation system can be fully adapted to the actual system (Table 2).

## 6. Examples and Results of the Analysis

Miner cost control is one of the important tasks of mining production. Through more accurate miner cost forecasting and control, parameters and mining parameters of the mine blocks are adjusted economically and reasonably, the personnel are arranged, and the personnel costs are reduced to improve results and benefits. The cost of mining personnel is closely related to the entire mining system and is affected by ventilation, drainage, transportation, and mining processes. The factors that affect the cost of mining personnel interact in a complex manner. Due to the complexity of the system, it is difficult to use traditional methods to build accurate and complete prediction and control models.

### 6.1. Mining Equipment

The equipment used in the mine development includes powdered ammonium nitrate explosive, light oil, detonating cords, explosive tubes, and detonators. The prices are shown in Table 3.

### 6.2. Mining Technology

When mining, the parameters of the mining process mainly include explosive unit consumption, row spacing, hole bottom distance, and collapse steps. Based on the theoretical and experimental research on the blastability evaluation of metal ore and the optimization of deep hole excavation parameters of the in-pit excavation sites, these parameters need to be considered in the optimal control model of production.

#### 6.2.1. Preliminary Determination of Explosive Unit Consumption

All test blast holes are artificially filled. According to relevant data and experience, the unit consumption q value of the funnel test explosive is taken as 3.25 kg/m^3^ and detonated at the bottom of the hole with an explosive tube detonator. After the explosive is filled, it will be severely blocked by taphole clay. After the blast hole is mined, the falling part of the laccolith around the funnel mouth is subtracted to determine the boundary of the funnel mouth. Take the blast hole as the center, take the radii *r* of nine funnels in different directions directly at 45°, use the average value as the radius *r* of the collecting funnel, to measure the actual minimum resistance cord *w*, and calculate the mining action index *n*. The funnel test data based on test statistics and calculation benchmarks are shown in Table 4.

The average radius *r* of the mining funnel obtained from Table 4 is 0.88 m, the average minimum resistance cord is 0.65 m, and the actual mining action index *n* = *r*/*w* = 1.38. The explosive consumption q value in actual standard unit is in turn calculated as 1.68 kg/m^3^ according to the formula of Polis Aube.

The number of columns in each unit consumption value experiment is all 10 columns, and the number of tests is four times. The number of columns corresponding to each detonation is two columns, two columns, three columns, and three columns. The detonation is delayed in milliseconds between the columns, and the time interval should not be less than 50 ms.  Table 5 shows the mining test results when different explosives are consumed separately.

Synthesizing the analysis and summary of the mining effect of multiple experiments, the reasonable unit consumption range of the mining area is 0.82–0.88 km/m^3^, and the unit consumption value is set to 0.86 km/m^3^ in the mining design. The actual unit consumption is controlled within the range of 0.82–088 kg/m^3^. The effect after mining is ideal, and the volume fraction is low (3%–25%). Afterwards, its impact on the construction is very small.

#### 6.2.2. Selection of the Distance between the Row Spacing of Fan-Shaped Deep Hole and the Hole Bottom

In the collapse of mining place, the interval between the fan-shaped deep holes is the minimum resistance line, which is usually determined by the diameter of the hole, the characteristics of the ore, the power of the explosive, and the degree of rock fragmentation. The distance between the bottom of the hole is the vertical distance between relatively shallow hole bottom and the deep blast holes. The blast hole density factor is the ratio of the bottom hole distance to the minimum resistance line, that is,

(17) $$\begin{array}{c} m=\frac{a}{w}, \end{array}$$

where *m* is the blast hole density coefficient; *A* is the bottom hole distance, *m*; *w* is the selection of the minimum resistance line.

The three parameters *m*, *a*, and *w* directly determine the hole density of the blast hole. The minimum resistance line reflects the density of the hole web between columns, and the bottom hole distance reflects the hole web density of the deep holes in the column, and the blast hole density coefficient reflects their mutual relationship. Whether the selection of these three parameters is correct will directly affect the economic and technical indicators in the mining process.

Combining the experience of various metallurgical mines, the blast hole density coefficient can be *m* = 1.0∼2.0. The relationship between the minimum resistance line *w* and the blast hole diameter *d* can be selected for reference from the actual data of the relevant mine. The value of the minimum resistance line used in mines is roughly as shown in Table 6 [13–15].

After the previously mentioned analysis, the design unit consumption is 0.85 kg/m^3^, and the actual unit consumption is mining tests with different distances and intervals in the range of 082–087 kg/m^3^. In the test, the hole bottom distances are divided into five groups, namely, 1.8 m, 2 m, 2.3 m, 2.4 m, and 2.5 m, respectively. Each group corresponds to seven kinds of intervals, 14 m, 15 m, 16 m, 18 m, 19 m, 20 m, and 21 m, respectively. The test site is located on the 2280 floor on the reexcavation channel of no. 23–25 detection line and the no. 19 detection line. Part of it is arranged on the return way of the no. 19 exploration line on the 2265 floor.

After mining, the mining effect records and analysis of seven different intervals are performed corresponding to five different hole bottom spacings. As the hole bottom distance and discharge interval increase, the impact of front row mining on the rear row of blast holes becomes more and more serious. The blast holes in the back row are blocked and misaligned more and more. The destruction of the eyebrow line gradually became apparent. The ceiling and the two groups will also be increased if they are missing. Obviously, the progress of the next mining project has slowed down. In the case of a certain hole bottom distance, as the cannon hole density coefficient increases, the volume rate after mining gradually decreases. If the big blast hole density coefficient increases to a certain range, a larger volume rate will be maintained. The relationship is shown in Figure 5.

Considering the comprehensive mining effect and project progress, the reasonable row spacing is 1.6–1.8 meters, and the reasonable hole bottom distance is 2–22 meters.

#### 6.2.3. Determination of the Step Pitch of Ore Caving

According to the results of multiple mining tests and the determination of the loss of ore drawing poverty, if two roads are used for collapsed mines simultaneously, the step distance of collapsed mines should preferably be three rows in each direction; that is, the stepped distance of collapsed mines is about 53 m. When a one-way road falls into a mine, the collapsed mines steps are preferably four columns per road. In other words, the collapsed mine step is about 7 meters.

Through a large number of field mining tests, mining parameters can be selected from Table 7.

### 6.3. Design of Wireless Communication Network

Compare the ratio of the amount of ore mined at one time to the cost of material used for mining 1 m^3^. The price performance ratio is considered as a measurement index, and cost performance is used as the output point of the model. In this way, the cost of equipment and personnel required for the volume of ore of the mining unit and the mining parameters are considered as the influencing factors of the system. This neural network model has nine input nodes. *Influence*. In other words, the model has nine input nodes. Due to the cost performance as the output of the model, the model has only one output node.

We collected a total of 20 learning samples, as shown in Table 8.

The first nine items in Table 6 are the input factors of the learning sample, and the last item is the output quantity. Use the samples in Table 8 to train the network. Before training, you should normalize the data not in [0, 1].

The model training, prediction, and appropriate program design calculations are carried out,. The model accuracy during training is 0.001, and the learning step is selected as 0.05. After 17 repetitions, the accuracy reached the requirement and the training was completed.  Figure 6 shows the error variance curve during model training. At this point, the connection weight of each node of the model has been determined. The same type of samples can be predicted at any time.

According to the range of mining equipment and mining process parameters, each element of the model is valued using interval intensive scanning technology in turn, which is used as the prediction sample of the model. Due to the large number of input factors and prediction samples, in order to ensure the comprehensiveness of the prediction samples, a computer is used to obtain values for the nine elements in sequence. Unsolicited data is automatically deleted. The selected prediction samples can be directly input into the model for prediction, and the performance-to-price ratio of all prediction samples can be obtained.  Table 9 shows the results of the inverse normalization after the prediction of the seven groups of prediction samples of the model.

According to the prediction results in Table 9, the deviation between the prediction and the actual situation is relatively small, and the prediction and actual results of the third and seventh groups are relatively high. Multiple production practices and wireless communication networks are combined to predict and control the cost of miners. This lead mine uses the best mining parameter values of the collapse method without sill pillar division. The explosive unit consumption is 0.87 kg/m^3^, the row spacing is 1.76 m, the hole bottom distance is 2.2 m, and the collapse step is 5.26 m. At this time, the actual price ratio of development reaches 33.78/yuan, which meets the production requirements.

## 7. Conclusions

In this paper, experiments on the budget and control of the cost of mining workers by wireless communication network technology have been carried out to prove that the characteristics of sandstone deposits are used to optimize the data, and the budget and control model of the cost of mining workers through wireless communication network technology are summarized. The method can accurately improve the mining work, guide the new direction of the mining design work, and provide favorable experience and data for mining similar mines.

## Figures and Tables

**Figure 1:** Cost network of mining personnel.

**Figure 2:** Membership function curve.

**Figure 3:** Mine development engineering drawing (partial).

**Figure 4:** The process of the cost control system for underground mining personnel.

**Figure 5:** The relationship charts between the blast hole density coefficient and the yield rate of large lumps.

**Figure 6:** Training error curve.

**Table 1:** Distribution of personnel in branches.

Branch	Wind resistance *R*_*j*_	Personnel *Q*_*j*_	Position of personnel	Structure placement
1	0.34	35.35		
2	0.41	37.02		
3	0.54	18.02		Allowable
4	0.91	20.02		
5	1.43	17.02	Allowable	Allowable
6	1.66	17.35		
7	0.22	35.02	Allowable	
8	0.17	37.35	Allowable	Allowable
9	0.01	72.25		

**Table 2:** The modular structure of cost control for mining personnel.

Serial number	Module name	Module content	Module role
1	Mining equipment	Shearers, supports, roadheader, etc.	Used for selection and layout of equipment
2	Transportation equipment	Mine carts, belt conveyors, transfer conveyor, mine carts tippers, scraper conveyors, etc.	
3	Lifting equipment	Main and auxiliary shaft hoists, cages, small winches, etc.	
4	Ventilation equipment	Fans, dampers, air ducts, etc.	
5	Drainage equipment	Water pump, pipeline, drain, sump pit	
6	Underground personnel	Coal mining, tunneling, support personnel, maintenance personnel, management personnel, etc.	For personnel management
7	Laneway	Horizontal main alley, underground parking lot, transportation main alley, transportation dip entry, crossheading, etc.	Used for 3D dynamic visualization of underground engineering
8	Underground chamber	Coal bunker, gangue bunker, etc.	System layout
9	Main and auxiliary shaft	Main shaft, auxiliary shaft, air shaft	
10	Coal face	Comprehensive mining, general mining, etc.	Selection of coal mining method
11	Face of heading	Comprehensive mining, general mining, etc.	Selection of tunneling methods
12	Support module	Working face support module, laneway support module	Selection of support mode
13	Mine production cycle operation module	Cycle operations of coal mining, tunneling, auxiliary production, etc.	Selection of work organization form
14	Mine excavation plan	Layout drawing of underground mining, layout drawing of mining work surface, etc.	Base map of the simulation system layout
15	CAD module	CAD system, CAD library	Import and draw CAD drawings
16	JMP analysis module	System reliability analysis indicators, etc.	Analyze the reliability of the system
17	Auxiliary function	System maintenance and other module	Other auxiliary functions of the supplementary system

**Table 3:** Prices of mining equipment.

Composition	Price	Average price
Powdery ammonium nitrate explosive/(yuan/t)	4700∼7000	5500
Diesel/(yuan/L)	709∼760	728
Detonating cord/(yuan/m)	51∼59	55
Nonel/(yuan/m)	10∼16	126
Detonator/(yuan/send)	84∼94	87

**Table 4:** Mining funnel test parameters.

Blast hole number	Explosion load (kg)	Loaded length (m)	Blockage length (m)	Funnel radius (m)	Design minimum resistance line (m)	Actual minimum resistance line	Mining effect evaluation	Data selection
1	087	04	05	084	065	066	Uniform lumpiness	Reserve
2	087	04	05	088	065	068	Uniform lumpiness	Reserve
3	087	04	05	—	065	—	Rushing stone	Reject
4	087	04	05	085	065	062	Uniform lumpiness	Reserve
5	087	04	05	074	065	073	Size of lump	Reject
6	087	04	05	118	065	055	Many chunk and fragment	Reject

**Table 5:** Mining test results of different explosive unit consumption.

Unit consumption/kg/m3	Row spacing (m)	Hole bottom distance (m)	Mining effect	Open wiring condition	Top board situation	Two side-wall situation	Rear blast hole situation
091–095	16	20	Overgrind of ore	Damaged severely	Lots of falling lumps and pumice	More slanting side-wall	Serious blocking of holes and dislocation
086–091	16	20	Small lumpiness, partly fine ore	Small damage	More pumice	Less slanting side-wall	More plugged holes, less dislocation
082–086	16	20	Uniform lumpiness, less fine ore	Less damage	Partial pumice and falling lumps	Less slanting side-wall	Less plugged holes and dislocation
075–082	16	20	Uneven lumpiness, high lump rate	Less damage	Less pumice and falling lumps	Rarely slanting side-wall	Occasionally plugged or misplaced

**Table 6:** Correspondence table of the relationship between the minimum resistance wire and the diameter of the blast hole.

Blast hole diameter (mm)	Minimum resistance line (m)	Blast hole diameter (mm)	Minimum resistance line (m)
50–60	12–17	60–85	18–28
60–70	15–22	90–125	26–45

**Table 7:** Mining parameters.

Mining parameters	Explosive unit consumption/(kg/m^3^)	Row spacing (m)	Hole bottom distance (m)	Ore drawing step pitch/row
Parameter value	0.83∼0.873	5∼1.9	1.8∼24	2∼5

**Table 8:** Learning sample.

Mining unit volume of ore mining equipment consumption					Operational parameter				Performance price ratio/(m^3^/yuan)
Powdery ammonia dynamite/(yuan/m^3^)	Diesel/(yuan/m^3^)	Detonating cord/(yuan/m^3^)	Nonel/(yuan/m^3^)	Detonator/(kg/m^3^)	Explosive unit consumption/(kg/m^3^)	Row spacing/m	Hole bottom distance/m	Ore drawing step pitch/row	
457	50	235	39	53	85	170	20	4	2672
435	48	224	3	42	82	172	21	4	3128
459	49	228	32	45	85	172	20	2	2693
471	51	265	33	46	87	16	19	2	250
444	48	225	30	41	82	166	21	3	307
453	49	235	34	48	84	171	20	2	2579
464	50	230	33	46	86	171	22	4	2930
455	49	228	36	50	84	169	19	3	2155
449	48	217	34	47	83	178	22	2	2740
463	50	228	31	43	86	168	21	3	2832
451	47	223	30	42	83	176	20	2	2809
463	50	240	31	44	86	171	22	3	3224
464	50	226	38	44	86	177	21	3	3672
454	49	236	29	41	84	164	21	4	3079
460	46	215	32	42	85	176	21	3	3284
455	49	238	33	45	84	19	22	3	2915
461	50	246	31	43	85	178	22	3	3332
460	49	244	34	47	85	167	2	4	2816
447	48	237	29	41	83	166	21	4	3556
445	49	225	31	43	82	173	21	2	3166

**Table 9:** Model prediction results.

Number	Mining unit volume of ore mining equipment consumption					Production process parameters				Performance price ratio	
	Powdery ammonium nitrate/(yuan/m^3^)	Diesel/(yuan/m^3^)	Detonating cord/(yuan/m^3^)	Nonel/(yuan/m^3^)	Detonator/(kg/m^3^)	Explosive unit consumption/(kg/m^3^)	Row spacing/m	Hole bottom distance/m	Ore drawing step pitch/row	Predicted	Actual
1	459	51	241	40	53	86	161	21	5	2735	2690
2	459	48	223	31	41	85	170	21	3	3023	3071
3	459	48	228	33	45	86	176	22	4	3293	3374
4	459	49	230	35	43	85	165	21	3	3123	3141
5	471	49	238	34	46	88	176	22	4	3009	3034
6	464	51	264	33	45	86	18	22	4	3021	2993
7	470	48	224	30	40	87	155	22	4	336	3357

## Data Availability

The labeled datasets used to support the findings of this study are available from the corresponding author upon request.
